The article "A Comparative Biomechanical Analysis of the Impact of Different Configurations of Pedicle-Screw-Based Fixation in Thoracolumbar Compression Fracture" was published in 2022. Journal: Appl Bionics Biomech.

# A Comparative Biomechanical Analysis of the Impact of Different Configurations of Pedicle-Screw-Based Fixation in Thoracolumbar Compression Fracture

**DOI:** 10.1155/2022/3817097

**Published:** 2022-02-23

**Authors:** Klaudia Szkoda-Poliszuk, Rafał Załuski

**Affiliations:** ^1^Department of Mechanics, Materials and Biomedical Engineering, Faculty of Mechanical Engineering, Wroclaw University of Science and Technology, Wroclaw, Poland; ^2^Department of Neurosurgery, Wroclaw Medical University, Wroclaw, Poland

## Abstract

The aim of this experimental study was to analyze the impact of applying different configurations of the transpedicular fixation system on selected mechanical parameters of the thoracolumbar spine under conditions of its instability (after simulated fracture). Five study groups were tested: physiological, with compression fracture of the vertebra, with two-segment fixation, with three-segment fixation, and with four-segment fixation. Each of the analyzed study groups was subjected to axial compression, flexion, and extension. Based on the conducted experimental tests, the mechanical parameters, i.e., stiffness coefficient and dissipation energy, were determined for all groups under consideration. The stiffness value of two-segment fixation is significantly lower than the physiological value (during flexion and extension). The use of long-segment fixation considered in two configurations (three- and four-segment fixation) may result in excessive stiffness of the system due to the high stiffness values achieved (approx. 25–30% higher than the physiological values in the case of compression and on average 60% higher in the case of flexion). The use of long-segment fixator design shows better results than short-segment fixation. Considering both biomechanical and clinical aspects, three-segment fixation seems to be a compromise solution as it saves the patient from more extensive stiffening of the spinal motion segments.

## 1. Introduction

According to statistics, fractures of the thoracolumbar spine (Th11-Th12-L1) account for almost 90% of all vertebral fractures and, moreover, approximately 50% of fractures are compression fractures of the Th12 or L1 vertebra [1–3]. The thoracic and lumbar segments differ in terms of the range of motion and structure of the individual vertebrae (resulting from the transmitted loads). The difference in the vertebral geometry is mainly manifested by the variable orientation of the facets of articular processes. In the zone of transition from one segment to another, the shape of the spine in the sagittal plane also changes. The existing thoracic kyphosis transitions into lumbar lordosis. All these factors affect the complex structure of this transition, increasing its instability and causing frequent injuries and mechanical damage.

In the case of vertebral fractures, surgical treatment of back injuries with implants has become standard clinical practice. However, it is often a major clinical problem and leads to many failures [4, 5]. This is mainly due to the different approaches of surgeons to the fixation of these fractures, particularly as regards the range of the stabilized spinal segment (number of stabilized spinal motion segments). Vertebral fractures in the thoracic and lumbar spine are usually stabilized by posterior short- or long-segment transpedicular fixation [3, 6, 7]. Current clinical practice is aimed at minimally invasive surgery. This technique saves the functional spinal units and thus significantly shortens the procedure [8].

However, there are discrepancies in the available literature regarding the behavior of the spinal segment subjected to loads under the conditions of discontinuity of the anterior column structure (compression fractures) and after its fixation [9–14]. According to a study conducted by Harms [9], damage to the vertebral body between the stabilized segments causes the fixator to take over approximately 90% of the load. Wang et al. [10] showed that transpedicular fixation of a vertebral fracture in the thoracolumbar spine does not provide sufficient stability, especially in the case of flexion. Based on available studies, fixation of fractures with displacement of bone fragments over two segments leads to many failures in surgical treatment [11–13]. The four-segment fixation, on the other hand, is characterized by a longer fixation area and greater limitation of the motor function compared to fixation of two adjacent segments [14]. The short-segment design allows for better clinical outcomes due to less fixation and less extensive surgery.

Therefore, experimental research may help to better understand the behavior of the thoracolumbar spine stabilized with implants. The aim of this experimental study was to analyze the impact of applying different configurations of the transpedicular fixation system on selected mechanical parameters of the thoracolumbar spine under conditions of its instability (after simulated compression fracture).

## 2. Materials and Methods

Experimental tests were carried out on specimens collected from eight domestic swine aged 6–10 months and weighing 90–110 kg. Isolated specimens of the thoracolumbar spine (Th7-L5) were cleaned of the surrounding soft tissues, leaving intact intervertebral discs, ligaments, and articular joints as well as partially ribs and muscles. The test material was stored in double foil packaging at -20°C until testing. The specimens were thawed at room temperature for several hours prior to testing.

In order to determine the impact of using different configurations of transpedicular fixation on selected mechanical parameters, five study groups were tested (Figure 1). First, the physiological system (P) was tested. Next, a compression fracture of the Th12 vertebra (CF) was performed. Thoracolumbar Spine Injury Classification System (AO classification) is divided into 3 injury subgroups: A (compression injuries), B (tension band injuries) and C (translational injuries in any axis) which are successively divided into subtypes [15]. Moreover, literature data show that approximately 50% of all fractures are compression fractures of the Th12 vertebra [1–3], where only the vertebral body is damaged without damage to the posterior column. On this basis, the type of fracture A2 was selected, which is a surgical treatment. The compression fracture type A2 was simulated in physiological specimens by an appropriate incision of the vertebral body (V-shape, as in the studies by Wang et al. [10]), to represent the effect of formation of this fracture and its morphology. A compression fracture is defined as a decrease in the height of the vertebral body during which it collapses. Hence, to simulate such a fracture, in experimental studies, it was decided to resect a large part of the vertebral body in its anterior region (approximately 30% of the vertebral body). This allowed for the mapping of a significant lowering of the vertebral body, simulating its collapse.

Next, transpedicular fixation was performed in each of the damaged thoracolumbar segments in three configurations: two-segment fixation (S2—1 level above and 1 level below the compression fracture), three-segment fixation (S3—2 levels above and 1 level below the compression fracture), and four-segment fixation (S4—2 levels above and 2 levels below the compression fracture). These three types of fixation design were selected for the analysis as they are most frequently used in clinical practice in the surgical treatment of compression fractures.

The experiment used the SOCORE transpedicular fixation system by NovaSpine, inserting polyaxial pedicle screws into the spine specimens (30° range of motion of the head relative to the screw). The vertebral bodies of the thoracic spine were implanted with screws with a diameter of 5 mm and a length of 35 mm, while the vertebral bodies of the lumbar spine were implanted with screws with a diameter of 6 mm and a length of 40 mm. Pedicle screws were connected with rods, 5.5 mm in diameter and of variable length depending on the length of the stabilized segment. In order to verify correct implantation of the pedicle screws in the vertebral bodies (Th10, Th11, L1, and L2), each of the specimens of the thoracolumbar spine was diagnosed by X-ray in the sagittal and coronal planes.

The specimens were loaded with forces reflecting normal life activities. The loading was carried out using an MTS 858 MiniBionix testing machine. The prepared specimens were mounted in a purpose-built test rig fitted with two grips (upper and lower), in which vertebral bodies Th7 and L5 were clamped with eight cylindrically arranged screws (Figure 2).

In the first stage, each of the analyzed study groups was subjected to pure axial compression with the force ranging from 150 to 650 N [16, 17]. The maximum applied compression load, acting with the force of 650 N, corresponds to the load transmitted through the lumbar spine of an average adult, resulting from the weight of the trunk, head, and upper limbs [10, 18, 19]. In subsequent stages, flexion and extension of the spinal column were simulated in the angular range of 0 to 4°. The maximum flexion and extension angles were adopted based on the assumptions of Panjabi et al. [20]. Each of the analyzed study groups was subjected to 20 load cycles at a frequency of 1 Hz corresponding to the frequency of human gait. It was also assumed that the first 4 cycles corresponded to conditioning cycles due to the properties of hyperelastic soft tissues, i.e., intervertebral discs or ligaments, and the need for their preloading to stabilize the test system.

Based on the conducted experimental tests, the mechanical parameters, i.e., stiffness coefficient and dissipation energy, were determined for all five study groups. Assessment of the stiffness of the different transpedicular fixation configurations allowed to determine which of the variants best reflected the physiological stability of the spine. By measuring the stiffness, it was checked which type of stabilization had a better effect on restoring the physiological stiffness and thus indirectly on restoring the physiological stability of the spine column. Stability was defined in the context of the system stiffness assessment.

In the case of compression load, the axial stiffness coefficient (*k*) was determined from the force-displacement loading curve obtained for the test specimens. The axial stiffness coefficient was determined in the force range from 350 N to 550 N for the 20th load cycle because in this section, the curve slope was linear and the increase in displacement was directly proportional to the applied load.

In the case of loads simulating flexion and extension, the bending stiffness coefficient (*k*_*M*_) was determined from the torque-deflection angle loading curve in the deflection angle ranging from 1.5° to 3.5° for the 20th load cycle because in this section, the curve slope was linear and the increase in the deflection angle was directly proportional to the applied load.

Dissipation energy of the examined spine specimens, otherwise known as the damping ratio, was determined based on the obtained hysteresis loops by calculating the difference between the area under the loading curve and the area under the unloading curve. Dissipation energy (as a parameter characterizing nonlinear mechanical properties) is determined, among others, by the viscoelastic nature of the annulus fibrous [21, 22]. The use of the energy criterion allows the assessment of the damping in the spine column. This makes it possible to describe, using energy criteria, the process of changes that can lead to damage under the action of external loading.

### 2.1. Statistical Analysis

All the results obtained from experimental testing were statistically analyzed using Statistica 13.1 software (StatSoft Inc., USA). The results for the five analyzed study groups were presented in the form of means with standard deviations. The parameters describing the effect of the type of fixation on the behavior of the spinal structures were analyzed using the Kruskal–Wallis nonparametric test with Dunn's multiple comparison post hoc test. The Kruskal-Wallis test is a nonparametric alternative to the one-way analysis of variance, allowing to compare the distributions of more than two independent groups, whose size is at least three in each case. Dunn's test is a post hoc pairwise test for multiple comparisons of mean rank sums. The statistical analyses were performed at a significant level of *p* < 0.05.

## 3. Results

The axial stiffness coefficient (*k*) for the group of physiological specimens averaged 224.0 ± 51.3 N/mm. As expected, the fracture disturbed the transmission of loads through the spinal column and led to instability, as indicated by an approximately 20% decrease in the mean value of the axial stiffness coefficient (179.7 ± 52.0 N/mm) compared to the value obtained for the physiological system.

The use of transpedicular fixation resulted in an increase in the stiffness coefficient compared to the value obtained for physiological specimens. In the case of use of S2 fixation, the mean *k* was approximately 9% higher compared to the value obtained for the group of physiological specimens. The use of long-segment fixation (S3 and S4) caused a significant increase in the stiffness coefficient compared to the values obtained for physiological specimens. These values were greater by approximately 22% (274.5 ± 68.5 N/mm) and approximately 29% (289.9 ± 65.3 N/mm), respectively. The increase in the mean *k* coefficient between S3 and S4 fixation was insignificant and amounted to approximately 5%. The demonstrated values of stiffness between the examined fixation systems showed no statistically significant differences (*p* > 0.05) (Figure 3(a)).

During flexion, the bending stiffness coefficient (*k*_*M*_) for the group of physiological specimens averaged 14.4 ± 3.4 Nm/rad. It was shown that the fracture caused instability, as reflected by the mean stiffness coefficient lower by approximately 28% compared to the value obtained for the physiological system. The use of S2 fixation resulted in decreased stiffness compared to the value obtained for physiological specimens. The mean stiffness coefficient was almost 41% lower than that obtained for physiological specimens (Figure 3(b)). On the other hand, the use of long-segment fixation (S3 and S4) caused a significant increase in the stiffness coefficient compared to the values obtained for physiological specimens. These values were greater by approximately 73% and approximately 49%, respectively.

In addition, statistically significant differences were demonstrated between the values obtained for the specimens with the Th12 vertebral fracture and the specimens treated with S3 fixation (*p* = 0.03). There were also statistically significant differences between S2 and S3 fixation (*p* = 0.009) as well as between S2 and S4 fixation (*p* = 0.04).

During extension, the stiffness coefficient *k*_*M*_ for the group of physiological specimens was higher by approximately 1.5 Nm/rad than the value obtained for the group of specimens with fracture (Figure 3(c)). The use of S2 fixation resulted in an approximately 41% decrease in the stiffness coefficient compared to the value obtained for physiological specimens. On the other hand, the use of long-segment fixation (S3 and S4) caused, as in the case of flexion, an increase in the stiffness coefficient (by approx. 29% and approx. 8%, respectively) compared to the values obtained for physiological specimens. Statistically significant differences were found between the values obtained for the specimens with S2 fixation and the values obtained for the group with S3 fixation (*p* = 0.009).

Analysis of the results of dissipation energy obtained for the axial compression showed that the mean damping energy of the examined spine specimens was 125.2 ± 23.2 mJ (Table 1). The greatest loss of dissipation energy was obtained for the group of specimens with the fracture of the vertebra. This value was greater by approximately 22% compared to the value obtained for physiological specimens. The lowest dissipation energy was obtained for the S4 fixation system. Statistically significant differences were found between the specimens with the fracture of the Th12 vertebra and those treated with four-segment fixation (*p* = 0.003).

During flexion, the mean damping energy of the examined physiological spine specimens was equal to the value obtained for the specimens with a fracture. The smallest loss of dissipation energy was obtained for the group of specimens treated with S2 fixation. This value was lower by approximately 32% compared to the value obtained for physiological specimens. It was also noticed that dissipation energy for the specimens with S3 fixation was slightly higher (by approx. 3.5 mJ) than the value obtained for the group with S2 fixation. The highest values of dissipation energy were obtained in the case of S4 fixation. No statistically significant differences were found between the analyzed study groups.

It was shown that during extension, the mean damping energy of the examined physiological spine specimens was practically equal to the value obtained for the specimens with a fracture. The values obtained for all three fixation configurations ranged from 23.5 to 26.2 mJ. The lowest loss of dissipation energy was obtained for the group of S4 specimens, and this value was smaller by approximately 48% compared to the value obtained for physiological specimens. No statistically significant differences were found between the analyzed study groups.

## 4. Discussion

The analysis of the obtained results showed a relationship between the stiffness coefficient and dissipation energy obtained for a given load case. An increase in the stiffness coefficient caused a decrease in the dissipation energy. The use of a more rigid system for long-segment fixation dampened less energy due to the fact that the acting load was transmitted mainly by the fixator and not by the system of intervertebral discs and ligaments with hyperelastic properties. A decrease in the stiffness coefficient increased dissipation energy, which in turn was probably related to the fact that the system needed more energy to resist the force while maintaining the original properties.

The high values of the standard deviation presented in Table 1 and in Figure 3 result from the dispersion of the obtained results around the mean. The wide dispersion of the results may be due to the variability in individual characteristics of the analyzed research objects, i.e., variability in the geometry of the vertebrae or variability in the inclination angles of individual segments of the spine. The dispersion of the results around the mean may also be caused by variability in the age (ranging between 6 and 10 months) and weight (ranging between 90 and 110 kg) of the swine used to collect the test specimens. The high standard deviations may also be due to the length of the test spine segment (Th7-L3).

It was also observed that in the case of Th12 vertebra fracture, the stiffness coefficient decreased for the compressive and bending loads and was significantly lower that the stiffness obtained for the physiological system. However, during extension, stiffness was similar to the physiological group and the group of vertebral fractures. This demonstrates that articular processes transmitted a significant part of the load during extension and fractures of the vertebra were not able to significantly disrupt the load transfer mechanism.

Based on the conducted experimental tests, it was shown that during flexion and extension, the stiffness coefficient obtained for S2 fixation was significantly lower than the physiological value, which in practice negates the usefulness of this solution because the fixator does not perform its function. This can be explained by the fact that fixation of the S2 segment is not able to completely prevent displacements in the area of the damaged vertebra, which is also indicated by the authors of other research studies [10, 14, 23]. Wang et al. [10] analyzed shorter specimens of the thoracolumbar spine (Th12-L3) for axial compression (250 N) and observed a similar relationship. The axial stiffness coefficient for the group of physiological specimens averaged 453 ± 58 N/mm. Due to the fact that shorter specimens of the thoracolumbar spine were analyzed, the values obtained by Wang et al. [10] are higher than the value obtained in this study (224 ± 51 N/mm). In the case of the use of S2 fixation, the mean stiffness coefficient was lower compared to the value obtained for the group of physiological specimens (170 ± 25 N/mm for 1/3 vertebral body injury). When comparing the value obtained by Wang et al., it was smaller than in this study (244 ± 69 N/mm). Elmasry et al. [23] analyzed the stiffness at the T12-L2 junction for flexion and extension (pure moments 7.5 Nm). Due to the fact that a shorter numerical model of the thoracolumbar spine was analyzed, the values obtained by Elmasry et al. are also higher than the value obtained in this study.

The analysis of the obtained results showed that S4 fixation can give better results than S2 fixation. It was noticed that during flexion and extension, the values of the stiffness coefficient obtained for S4 fixation were closest to the values obtained for the physiological system. However, the use of S4 fixation resulted in significantly longer time of surgery. On the other hand, the S3 configuration allows for a less extensive fixation of the spine compared to S4. From the functional point of view, the shorter the fixation time, the better for the patient. Moreover, to obtain good clinical effects of treatment, it is crucial to reduce kyphosis and restore the correct sagittal position of the spine, which can be ensured by S3 fixation relative to S2 fixation [8].

McDonnell et al. [24] and Bolesta et al. [25] also observed in experimental studies that S2 fixation cannot reflect the physiological stability of the thoracolumbar spine. On the other hand, the results presented in the same studies indicate the achievement of immediate stability of the damaged spinal segment with the use of S4 fixation and the obtained greater stiffness compared to the physiological specimens. Nonetheless, Bolesta et al. [25] emphasize that in the case of S2, it is worth considering a configuration with two additional screws inserted into the damaged vertebra. The morphology of the fracture, however, often prevents the use of this solution, for example, in the case of a fracture of the vertebral epiphysis. In this case, an alternative is to use S3 fixation. Despite including a larger number of stabilized vertebrae than S2 fixation (even with an additional screw in the area of the fractured vertebra), provides an adequate fracture reduction and restoration of the spinal curvature. According to clinical practice, there is no indication for the use of an additional screw in a compression fracture (Sun et al., 2016). This strategy may be used in less unstable scenarios, such as in burst fractures, especially in distraction or translation injuries. The inclusion of screws at the fracture level prolongs the surgical treatment time, which is a disadvantage in minimally invasive surgery. McDonnell et al. [24] emphasize that pedicle screws at the fracture level did not improve stability in the short- or long-segment fixation.

Elmasry et al. [23] and McDonnell et al. [24] both report that long-segment fixation has higher stiffness and restricts range of motion better than short-segment fixation. However, according to Elmasry et al. [23], inclusion of screws at the fracture level in long constructions, paradoxically, decreased stiffness of the fixation, as the intermediate screw was postulated to act like a pivot.

Sun et al. [26] reported the results of 69 patients with thoracolumbar burst fractures treated with a short-segment fixation (34 patients) versus short-segment fixation with screws at the fracture level (35 patients). Both groups had similar preoperative characteristics (clinical and radiological). While no differences in the outcome of the 2 groups were documented, short-segment fixation had the advantages of less operative time, blood loss, and hospitalization time. They concluded that short-segment fixation might be sufficient to treat burst fractures surgically, regardless of the inclusion of the fractured vertebra.

The obtained results allowed to assess which fixation configuration can best restore the physiological stiffness. The test results showed the following:

- S2 fixation can reflect the physiological stiffness in the case of compression because the obtained value is the closest to that obtained for the physiological case
- During flexion and extension, the stiffness value of S2 fixation is significantly lower than the physiological value, which in practice negates the usefulness of this solution because the fixator does not perform its function
- During both compression and flexion, the use of long-segment fixation considered in two configurations (S3 and S4) may result in excessive stiffness of the system due to the high stiffness values achieved (approx. 25–30% higher than the physiological values in the case of compression and on average 60% higher in the case of flexion)
- During loading simulating extension, the greatest excessive stiffness may be caused by S3 fixation due to the highest stiffness coefficient while S4 fixation works best in the process reflecting the physiological stiffness

Summarizing the results obtained from experimental testing, it can be said that fixation of the Th12 vertebra fracture over two segments does not provide adequate stability to the spinal column during flexion and extension. On the other hand, the use of long-segment fixation for this type of fracture may lead to excessive stiffness of the considered spinal segment. Consequently, this may contribute to increased mobility of the segments immediately adjacent to the implantation site, raising the risk of increasing curvature of thoracic kyphosis, which may result in the breakage or loosening of transpedicular screws [27, 28]. Breakage and loosening of the transpedicular screw are the most common complications that affect spinal stability. Currently, numerous experimental and numerical studies are conducted to analyze the effect of bending and pulling out of pedicle screws [29, 30]. Considering both biomechanical and clinical aspects, S3 fixation seems to be a compromise solution as it saves the patient from more extensive stiffening of the spinal motion segments.

### 4.1. Limitations of the Study

Animal-derived preparations are commonly used as research models to replace human preparations (sectional preparations) in experimental research. Due to the limited availability of human preparations, scientists are constantly looking for a representative animal model that reflects the biomechanics and anatomy of the human spine. Therefore, in experimental studies, the porcine spine was used as a physiologically correct preparation, unchanged under the influence of deformation.

The lumbar spine of porcine is characterized by a high anatomical and structural similarity to the lumbar spine of humans, mainly in terms of geometric parameters of the vertebrae [31, 32]. Busscher et al. [32] studied the anatomy of human and porcine spine segments and concluded that porcine spine models are representative for researching human spine anatomy. Busscher et al. also found that the biomechanical behavior of the human lumbar spine is comparable with the low thoracic and lumbar porcine spine, which implies that the porcine model can be used as a valid model for investigation. They based on measurements of the geometry of the human and porcine spine, showing that the mean total spine length differed by 0.1 mm between the human and porcine spines (respectively, 569.4 ± 17.67 mm and 569.5 ± 16.19 mm).

It was also proved that the heights of human and porcine vertebrae in individual sections of the spine were similar to each other. By comparing the width and height of the spinal canal in individual vertebrae between the human and porcine spine, it can be concluded that porcine vertebrae can be a representative model when testing fixation system techniques. In particular, it is noted that the width of the spinal canal of porcine vertebrae indicates remarkable similarity to the same parameter in human vertebrae [33, 34]. The human spine shows less cervical lordosis (20.1°) and more pronounced thoracic kyphosis (34.5°) and lumbar lordosis (29.2°). In the porcine spine, these values are, respectively, 43.8° (cervical lordosis), 15.6° (thoracic kyphosis), and 7.9° (lumbar lordosis).

Despite the fact that differences in the curvature of individual sections of the spine are observed when comparing the dimensions of the spinal canal in individual vertebrae between the human and porcine spine, the literature shows that porcine vertebrae can be a representative model when testing fixation system techniques [32, 33].

Additionally, while developing the testing protocol used in this study, it was observed that tests performed on such long segments of the spine (Th7-L5) sometimes led to their buckling during loading with compressive force. It has been noticed that the danger of loss of stability is not due to simulated trauma but due to the lack of active support of the muscular system. Therefore, in order to eliminate the undesirable phenomenon of buckling, the costovertebral joints (connecting the proximal end of the ribs with their corresponding thoracic vertebrae) and muscles surrounding the isolated specimens were not removed. Moreover, the limitation of the number of load cycles was also applied for each tested case in order to minimize the risk of loss of stability, which could consequently (in some cases of the applied stabilization) lead to a second loss of stability.

## 5. Conclusion

Our findings can be used in studies using human cadavers and subsequently in clinical research related to the introduction of new implant solutions for the fixation of thoracolumbar spine injuries. Due to the anatomical similarity (the animal model to human dissection preparations), it can be suggested that the simulated type of the fracture and its influence on the obtained mechanical parameters after stabilization also occur in the case of the human spine. The cognitive aspects also include the fact that the obtained mechanical parameters can be used to implement complex numerical models of the spine.

It should be emphasized that experimental studies on animal models are more accurate than numerical simulation. Experimental studies reflect the variability of material properties to a greater extent, especially when it comes to spine structure. The spine is a complex structure with nonlinear material properties, especially the intervertebral disc, which has viscoelastic properties. Often, to optimize the numerical simulations, simplifications are introduced in the model. The simplifications mainly relate to among others the material parameters or boundary conditions. This is a limitation of the numerical analysis carried out.

The experimental results of the biomechanical study allow us to draw the following conclusions:

- The use of long-segment fixator design shows better results than short-segment fixation
- Short-segment fixator design does not provide sufficient stability, especially in the case of flexion. The use of this type of fixator configuration may not provide adequate stiffness, thereby resulting in excessive mobility of the transitional zone
- The use of S3 fixation allows to optimize the biomechanical and clinical conditions in a situation where it is impossible to insert a screw into a fractured vertebra

## Figures and Tables

**Figure 1:** Considered configurations of the posterior spinal fixation system: (a) physiological (P), (b) with compression fracture of the Th12 vertebra (CF), (c) with two-segment fixation (S2), (d) with three-segment fixation (S3), and (e) with four-segment fixation (S4).

**Figure 2:** Specimen in the loading system: (a) axial compression; (b) flexion/extension.

**Figure 3:** Stiffness coefficient for (a) axial compression, (b) flexion, and (c) extension.

**Table 1:** Mean values of dissipation energy (∆*E*) with standard deviations (SD) for the considered configurations.

Loads	Considered configurations				
	P	CF	S2	S3	S4
	Δ*E* (mJ)				
Compression	125.2 ± 23.2	152.7 ± 31.1	123.0 ± 25.6	106.2 ± 21.4	97.5 ± 21.6
Flexion	32.1 ± 14.1	32.7 ± 13.2	22.1 ± 7.4	25.7 ± 8.3	30.1 ± 5.9
Extension	41.2 ± 16.3	42.4 ± 16.1	23.5 ± 7.7	26.2 ± 10.4	21.4 ± 7.8

## Data Availability

The data used to support the findings of this study are included within the article.
